# Clinical Observation of Reduning Combined with Recombinant Human Interferon *α*-2b in the Treatment of Children with Viral Pneumonia

**DOI:** 10.1155/2022/1739561

**Published:** 2022-06-14

**Authors:** Zhuangzhuang Li, Lingling Xie, He Wang, Shugen Wang, Jinguang Wu

**Affiliations:** Department of Pharmacy, Cangzhou Central Hospital, Cangzhou 061000, Hebei, China

## Abstract

**Purpose:**

To observe the clinical efficacy of Reduning injection combined with recombinant human interferon *α*-2b spray in the treatment of children with viral pneumonia.

**Methods:**

A total of 200 children with viral pneumonia over 2 years old who were admitted to the Pediatrics Department of the Cangzhou Central Hospital from September 2018 to November 2020 were recruited and randomized into the control group and observation group at a ratio of 1 : 1, with 100 cases in each group. The children in the control group were given recombinant human interferon *α*-2b spray, and the children in the observation group were given Reduning injection on the basis of the control group. The clinical symptoms and signs, clinical efficacy, levels of inflammatory mediators, and drug safety were compared between the two groups.

**Results:**

The *t*-test results showed that the disappearance time of body temperature, respiratory rate, pulmonary rales, and cough in the observation group was significantly shorter than that in the control group. The chi-square revealed a significantly higher total effective rate in the observation group vs. the control group. After treatment, the levels of IL-1, IL-6, TNF-*α*, and CRP in the two groups were lower than the corresponding values before treatment, and greater reduction was observed in the observation group in relative to the control group (both *p* < 0.05). The two groups have a similar safety profile.

**Conclusion:**

Reduning combined with recombinant human interferon *α*-2b produces a remarkable effect in the treatment of children with viral pneumonia, and it ameliorates clinical symptoms and reduces inflammatory response with a good safety profile.

## 1. Introduction

Viral pneumonia is a common respiratory tract infectious disease in children [1]. Due to the wide spread of pathogenic bacteria (such as droplets and direct contact), fast transmission, and sudden onset, it is prone to multisystem diseases complicating with the heart and brain in severe cases, seriously threatening the growth and development of children [2, 3]. Respiratory syncytial virus pneumonia is common in infants and young children under the age of 2 and often presents with symptoms and signs such as wheezing, dyspnea, and pulmonary fine moist rales. At present, the incidence of viral pneumonia in children is on the rise [4, 5].

Clinically, the absence of specific drugs for children with viral pneumonia requires symptomatic and supportive treatment of antiviral drugs and antibiotics [6]. Among them, aerosol inhalation of recombinant human interferon *α*-2b is used to treat viral respiratory tract infections, with merits of direct action on the respiratory mucosa, strong target properties, and good effectiveness and safety profiles [7]. Studies have shown that interferon *α*-2b has a dual mechanism of antiviral and immune regulation. On the one hand, interferon *α*-2b activates the JAK/STAK signal transduction pathway by binding with type I interferon receptors on the cell surface and eventually activates about 300 kinds of interferon stimulation genes to synthesize a large number of antiviral proteins. It plays an antiviral role against different targets in the life cycle of viruses. On the one hand, interferon *α*-2b plays an antiviral role by enhancing the cellular immune function [8, 9].

Traditional Chinese medicine (TCM) plays an important role of viral pneumonia in children. In TCM theory, children' viscera is delicate, the shape and qi are not filled, and the self-regulated functions of cold and warmth are not formed, giving rise to invasion of external pathogens, phlegm-damp stagnation, obstructed airways, and accumulated heat and toxin. Considering this, the treatment should be conducted based on dispersing the lung and lowering qi, eliminating phlegm, and relieving dyspnea [10, 11]. Reduning injection, a pure TCM injection, has the functions of clearing away heat, dispelling wind, and detoxification and is used to treat cough, upper respiratory tract infection, and acute bronchitis, with definite clinical efficacy [12]. In light of this, this study aimed to investigate the efficacy of Reduning injection combined with recombinant human interferon alpha-2b in the treatment of children with viral pneumonia.

## 2. Materials and Methods

### 2.1. Participants

Between September 2018 and November 2020, two hundreds viral pneumonia children who were admitted to the Pediatric Department of the Cangzhou Central Hospital were enrolled in the present study. All enrollments were randomized into the control group and observation group, with 100 cases in each group. The protocol in the study followed the relevant regulations of the Ethics Committee and were approved by the ethics committee of the Cangzhou Central Hospital.

### 2.2. Inclusion and Exclusion Criteria

Inclusion criteria were as follows: the children had symptoms such as fever, cough, shortness of breath and dyspnea, and lung rales; with signs of pneumonia on chest radiographs and low inflammatory mediators; in line with the diagnostic criteria for viral pneumonia in children by Practical Pediatrics; pneumonia virus antibodies positive; and visited a doctor within 48 hours of onset.

Exclusion criteria were as follows: children with nonviral pneumonia; children with contraindications to this drug; and children with severe illness.

### 2.3. Interventions

After admission, both groups were given routine symptomatic and supportive treatment, and the control group was given recombinant human interferon alpha-2b (produced by Anhui Anke Bioengineering (Group) Co., Ltd., approval no.: S20000013, specification: 3 million IU/tube) that was mixed with normal saline to a total volume of 2 mL, via aerosol inhalation, 2 times a day with the interval >6 hours. The observation group was given Reduning injection (Jiangsu Kangyuan Pharmaceutical Co., Ltd., approval no.: Z20050217, specification: 10 mL/piece) intravenously on the basis of the treatment in the control group; for children aged 3–5 years, it was given via intravenous drip by adding less than 10 mL to 0.9% 50–100 mL sodium chloride injection at a drip rate of 30–40 drops/min; for children aged 6–11 years, it was given via intravenous drip by adding 10 mL/time to 0.9% 100–200 mL sodium chloride injection at a drip rate of 30–60 drops/min, once a day. A course of treatment in both groups was taken as 5–7 days.

### 2.4. Efficacy Observation and Evaluation Criteria

1. Clinical symptoms and signs: before treatment and within 1 week after treatment, the clinical symptoms and signs of the two groups of children were observed daily, including body temperature, respiratory rate, pulmonary rales, and cough.
2. Clinical efficacy: the clinical efficacy is categorized into cured (normal body temperature, respiratory failure, expectoration, and other symptoms completely disappear, and lung imaging examination shows that all the inflammatory areas are absorbed), markedly effective (basically, normal body temperature, respiratory failure, expectoration, and other symptoms are visible, and lung imaging examination shows that the inflammation area is basically absorbed), ineffective (fever, respiratory failure, expectoration, and other symptoms are not relieved, and lung imaging examination shows that the inflammation area is not absorbed); total effective rate = (cured + markedly effective)/total number of patients × 100%.
3. Inflammatory mediators: serum factors such as C-reactive protein (CRP) were detected by enzyme-linked immunosorbent assay before and after treatment.
4. Drug safety: the adverse reaction rates of the two groups were compared, including nausea, vomiting, dizziness, and rash.

### 2.5. Statistical Analysis

All data analyses were performed with SPSS 26.00. Measurement data were expressed as ($\bar{x}\pm s$) and processed using the *t*-test, while count data were expressed as % and examined via the *χ*^2^ test. The level of significance was set at *p* < 0.05.

## 3. Results

### 3.1. Comparison of General Data

In the observation group, there were 59 males and 41 females, the age was 2–10 (5.64 ± 1.75) years old, the course of disease was 1–8 (4.28 ± 1.32) days, and the body temperature was (39.7 ± 0.6)°C. In the control group, there were 57 males and 43 females, the age was 2–11 (5.91 ± 1.62) years, the course of disease was 1–9 (4.43 ± 1.53) days, and the body temperature was (39.6 ± 0.5)°C. The two groups presented good comparability in gender, course of disease, and body temperature (Table 1).

### 3.2. Comparison of the Disappearance Time of Symptoms and Signs

The disappearance time of body temperature, respiratory rate, pulmonary rales, and cough in the observation group was significantly shorter than that in the control group (all *p* < 0.001) (Table 2).

### 3.3. Comparison of Clinical Efficacy

The chi-square revealed a significantly higher total effective rate in the observation group vs. the control group (*p* < 0.05) (Table 3).

### 3.4. Comparison of the Levels of Inflammatory Mediators

Before treatment, there was no significant difference in the levels of inflammatory mediators between the two groups (*p* > 0.05). After treatment, the levels of IL-1, IL-6, TNF-*α*, and CRP in the two groups were lower than the corresponding values before treatment, and greater reduction was observed in the observation group in relative to the control group (both *p* < 0.05) (Table 4).

### 3.5. Comparison of Adverse Reactions

In the observation group, there were 3 cases of nausea and vomiting, 5 cases of dizziness, and 0 cases of rash; the control group had 4 cases of nausea and vomiting, 3 cases of dizziness, and 1 case of rash. Overall, the two groups have a similar safety profile, as given in Table 5.

## 4. Discussion

The high incidence of viral pneumonia in children is associated with the respiratory anatomy results such as short respiratory tract, narrow lumen, and weak ciliary motility in children [13, 14]. Children are susceptible to respiratory viruses, along with the incomplete immune system and poor immune memory and antigen presentation, resulting in repeated respiratory infections and pneumonia, with viral pneumonia more common [15]. Recombinant human interferon *α*-2b, a broad-spectrum antiviral drug, plays an important role in inhibiting cell proliferation and improving human immunity. Interferon is a group of low molecular weight glycoproteins produced by immune cells in response to a virus infection [16, 17]. In this regard, supplementing exogenous interferon can inhibit the proliferation of virus-infected cells, enhance immune regulation activity, mitigate the virus symptoms of pneumonia, and reduce inflammatory response [18]. With the progress of research, it is found that the drug resistance of most viruses will gradually increase, which will further cause adverse reactions during treatment and compromise the efficacy of treatment. In recent years, the treatment of integrated traditional Chinese and Western medicine has become a research hotspot. In the present study, we innovatively treat respiratory syncytial virus infection with integrated traditional Chinese and Western medicine and observe its efficacy [19].

Reduning injection, as a typical Western-made traditional Chinese medicine, is mainly composed of *Artemisia annua*, honeysuckle, and *Gardenia* [20]. Honeysuckle disperses wind-heat, clears heat and detoxifies, has anti-inflammatory and antiviral properties, promotes and restores the phagocytic ability of white blood cells, promotes lymphocyte transformation, and regulates immune function. *Gardenia* can conduct toxin down, eliminate the fire of Sanjiao, and enhance the detoxification effect of honeysuckle, and modern pharmacological research believes that it has anti-inflammatory, antiviral, cooling and antipyretic effects. *Artemisia* can relieve exterior syndrome, clear away the heat, and the main component of Artemisia annua has anti-inflammatory, antipyretic, analgesic, and immunity-enhancing effects, and artemisinin and artemether have the function of promoting the proliferation of spleen *T* lymphocytes, and exert direct effect in inactivating and inhibiting proliferation of influenza virus [21, 22].

This study showed that the body temperature, respiratory rate, pulmonary rales, cough disappearance time, and treatment efficiency of the observation group were significantly better than those of the control group, suggesting that the treatment of integrated traditional Chinese and Western medicine can exert synergetic effects to relieve the clinical symptoms. Additionally, the levels of inflammatory mediators IL-1, IL-6, TNF-*α*, and CRP in the observation group were significantly lower than those in the control group. As previously noted, serum CRP is an important indicator for diagnosing bacterial infection and demonstrates a positive correlation with the degree of infection [23]. All these indicate that the combined treatment leads to a milder pulmonary inflammatory factor response and lower serum CRP in children. More importantly, the two groups showed a similar safety profile in terms of the incidence of adverse reactions, suggesting an acceptable safety profile.

## 5. Conclusion

Recombinant human interferon *α*-2b combined with Reduning might be a promising alternative in the treatment of children with respiratory syncytial virus infection pneumonia by relieving the clinical symptoms of children, reducing inflammatory reactions, and driving down the adverse reactions. It has good safety and effectiveness profiles and thus merits clinical application.

## Figures and Tables

**Table 1:** General data.

	Observation group (*n* = 100)	Control group (*n* = 100)	*χ* ^2^/*t*	*P*
Gender			0.082	0.774
Male	59	57		
Female	41	43		
Age (years)	5.64 ± 1.75	5.91 ± 1.62	1.132	0.259
Disease course (days)	4.28 ± 1.32	4.43 ± 1.53	0.742	0.459
Body temperature	39.7 ± 0.6	39.6 ± 0.5	1.28	0.202

**Table 2:** Comparison of the disappearance time of symptoms and signs between the two groups ($\bar{x}\pm s$, days).

	*n*	Body temperature	Respiratory rate	Pulmonary rales	Coughing
Observation group	100	4.16 ± 0.53	1.62 ± 0.33	3.11 ± 0.91	3.77 ± 1.13
Control group	100	5.48 ± 1.27	3.75 ± 0.82	6.10 ± 1.87	6.73 ± 2.54
*t*		9.592	24.097	14.377	10.647
*P*		<0.001	<0.001	<0.001	<0.001

**Table 3:** Comparison of efficacy (*n*, %).

	*n*	Cured	Markedly effective	Ineffective	Total (%)
Observation group	100	20	73	7	93
Control group	100	15	59	26	74
*χ* ^2^					13.101
*P*					<0.001

**Table 4:** Comparison of the levels of inflammatory mediators ($\bar{x}\pm s$, pg/mL).

	*n*	IL-1		IL-6		TNF-*α*		CRP	
		Before treatment	After treatment	Before treatment	After treatment	Before treatment	After treatment	Before treatment	After treatment
Observation group	100	141.86 ± 5.86	88.34 ± 4.02^*∗*^	248.09 ± 5.37	98.91 ± 3.54^*∗*^	146.12 ± 7.73	86.54 ± 3.34^*∗*^	17.71 ± 2.33	3.02 ± 1.34^*∗*^
Control group	100	140.93 ± 5.72	110.73 ± 5.34^*∗*^	249.35 ± 6.07	108.11 ± 5.72^*∗*^	147.25 ± 8.32	100.61 ± 5.77^*∗*^	17.68 ± 2.18	4.97 ± 1.58^*∗*^
*t*		1.136	33.498	1.555	13.677	0.995	21.104	0.094	9.412
*P*		0.257	<0.001	0.122	<0.001	0.321	<0.001	0.925	<0.001

Compared to the corresponding values before treatment within the group, ^*∗*^*p* < 0.05.

**Table 5:** Comparison of adverse reactions (*n*, %).

	*n*	Nausea and vomiting	Dizziness	Rash	Total
Observation group	100	3	5	0	8
Control group	100	4	3	1	8
*χ* ^2^					0.13
*P*					0.718

## Data Availability

The datasets used during the present study are available from the corresponding author upon request.

## References

[1] Dandachi D., Rodriguez-Barradas M. C. (2018). Viral pneumonia: etiologies and treatment. *Journal of Investigative Medicine*.

[2] Gattarello S., Rello J. (2017). Severe viral pneumonia in adults: what is important for the ICU physician?. *Hospital Practice*.

[3] Yun K. W., Wallihan R., Juergensen A., Mejias A., Ramilo O. (2019). Community-acquired pneumonia in children: myths and facts. *American Journal of Perinatology*.

[4] Castagnoli R., Votto M., Licari A. (2020). Severe acute respiratory syndrome coronavirus 2 (SARS-CoV 2) infection in children and adolescents: a systematic review. *JAMA Pediatrics*.

[5] Chen X. B., Du S. H., Lu J. C. (2020). Retrospective analysis of 61 cases of children died of viral pneumonia. *Fa Yi Xue Za Zhi*.

[6] Ruuskanen O., Lahti E., Jennings L. C., Murdoch D. R. (2011). Viral pneumonia. *The Lancet*.

[7] Mulder K., Patel A. A., Kong W. T. (2021). Cross-tissue single-cell landscape of human monocytes and macrophages in health and disease. *Immunity*.

[8] Gao J., Zhao B. R., Zhang H., You Y. L., Li F., Wang X. W. (2021). Interferon functional analog activates antiviral Jak/Stat signaling through integrin in an arthropod. *Cell Reports*.

[9] O’Shea J. J., Plenge R. (2012). JAK and STAT signaling molecules in immunoregulation and immune-mediated disease. *Immunity*.

[10] Sun L., Wang D., Xu Y., Qi W., Wang Y. (2020). Evidence of TCM theory in treating the same disease with different methods: treatment of pneumonia with ephedra sinica and scutellariae radix as an example. *Evidence-Based Complementary and Alternative Medicine*.

[11] Sun Q., Yu H., Shang Y., Cao Y. (2021). Correlation analysis of chaige qinlian decoction and acupuncture combined intervention on prognosis of children with pneumonia. *Journal of Healthcare Engineering*.

[12] Cao C., Zhen Z., Kuang S., Xu T. (2020). Reduning injection combined with western medicine for pneumonia: a protocol for systematic review and meta-analysis. *Medicine*.

[13] Jeena P. M., Govender K., Parboosing R., Adhikari M. (2017). The significance of cytomegalovirus in children with pneumonia admitted for mechanical ventilation. *International Journal of Tuberculosis & Lung Disease*.

[14] Izadnegahdar R., Cohen A. L., Klugman K. P., Qazi S. A. (2013). Childhood pneumonia in developing countries. *Lancet Respiratory Medicine*.

[15] Erdem S. B., Can D., Girit S. (2018). Does atopy affect the course of viral pneumonia?. *Allergologia et Immunopathologia*.

[16] Lewczuk N., Zdebik A., Bogusławska J. (2019). Interferon alpha 2a and 2b in ophthalmology: a review. *Journal of Interferon and Cytokine Research*.

[17] Pandit A., Bhalani N., Bhushan B. S. (2021). Efficacy and safety of pegylated interferon alfa-2b in moderate COVID-19: a phase II, randomized, controlled, open-label study. *International Journal of Infectious Diseases*.

[18] Yang A., Yang C., Yang B. (2020). Use of hydroxychloroquine and interferon alpha-2b for the prophylaxis of COVID-19. *Medical Hypotheses*.

[19] Huang K., Zhang P., Zhang Z. (2021). Traditional Chinese medicine (TCM) in the treatment of COVID-19 and other viral infections: efficacies and mechanisms. *Pharmacology & Therapeutics*.

[20] Wang Z., Chen W., Li Y. (2021). Reduning injection and its effective constituent luteoloside protect against sepsis partly via inhibition of HMGB1/TLR4/NF-*κ*B/MAPKs signaling pathways. *Journal of Ethnopharmacology*.

[21] Zhang G., Li Y., Chen T. (2019). Comparative study of the efficacy and pharmacokinetics of reduning injection and atomization inhalation. *Biomedicine & Pharmacotherapy*.

[22] Xie F., Xie M., Yang Y. (2020). Assessing the anti-inflammatory mechanism of reduning injection by network pharmacology. *BioMed Research International*.

[23] Hu L., Shi Q., Shi M., Liu R., Wang C. (2017). Diagnostic value of pct and CRP for detecting serious bacterial infections in patients with fever of unknown origin: a systematic review and meta-analysis. *Applied Immunohistochemistry & Molecular Morphology*.

